The article "Impact of Physical Activity on Oxidative Stress Markers in Patients with Metastatic Breast Cancer" was published in 2021. Journal: Oxid Med Cell Longev.

# Impact of Physical Activity on Oxidative Stress Markers in Patients with Metastatic Breast Cancer

**DOI:** 10.1155/2021/6694594

**Published:** 2021-07-16

**Authors:** Lidia Delrieu, Marina Touillaud, Olivia Pérol, Magali Morelle, Agnès Martin, Christine M. Friedenreich, Pauline Mury, Armelle Dufresne, Thomas Bachelot, Pierre-Etienne Heudel, Béatrice Fervers, Olivier Trédan, Vincent Pialoux

**Affiliations:** ^1^Inter-University Laboratory of Human Movement Biology EA7424, University Claude Bernard Lyon 1, University of Lyon, Lyon, France; ^2^Department of Cancer and Environment, Léon Bérard Cancer Center, Lyon, France; ^3^Unité INSERM UA8, Centre Léon Bérard, Ministère des Armées, "Radiations: Défense, Santé et Environnement", Lyon, France; ^4^Department of Clinical Research and Innovation, Léon Bérard Cancer Center, Lyon, France; ^5^Department of Cancer Epidemiology and Prevention Research, Cancer Care Alberta, Alberta Health Services, Calgary, Alberta, Canada; ^6^Departments of Oncology and Community Health Sciences, Cumming School of Medicine, University of Calgary, Calgary, Alberta, Canada; ^7^Department of Medical Oncology, Léon Bérard Cancer Center, Lyon, France; ^8^Institut Universitaire de France (IUF), Paris, France

## Abstract

**Purpose:**

Regular physical activity (PA) can affect oxidative stress, known to be involved in carcinogenesis. The objective of this study was to evaluate the associations between a six-month PA intervention and oxidative stress biomarkers, PA, and clinical outcomes in patients with metastatic breast cancer.

**Methods:**

Forty-nine newly diagnosed patients with metastatic breast cancer were recruited for a single-arm, unsupervised, and personalized six-month walking intervention with activity tracker. PA level and PA fitness, plasma concentrations of DNA oxidation (8OhdG), lipid peroxidation (MDA), and protein oxidation (AOPP), plasma activities of superoxide dismutase (SOD), glutathione peroxidase (GPX), and catalase, plasma and leucocyte activities of myeloperoxidase (MPO) and NADPH oxidase (NOX), and clinical markers of tumor progression (RECIST criteria) were measured at baseline and after the six-month intervention.

**Results:**

GPX activity (+17%) and MDA (+9%) significantly increased between baseline and the end of the intervention. Changes in PA level and fitness were significantly positively correlated with changes in plasma GPX and significantly negatively with changes in NOX in the leucocytes. Plasma MDA was significantly higher (+20%) whereas plasma AOPP was lower (-46%) for patients with tumor progression or that died during the six months as compared to patients without progression.

**Conclusion:**

A six-month PA intervention may be potentially beneficial in metastatic breast cancer patients for enhancing antioxidant enzyme activity and decreasing prooxidant enzyme activity. Moreover, AOPP and MDA could also be favorable and unfavorable biomarkers, respectively, since they are associated with disease progression and fitness level in this population. This trial is registered with NCT number: NCT03148886.

The article "Impact of Physical Activity on Oxidative Stress Markers in Patients with Metastatic Breast Cancer" was published in 2021. Journal: Oxid Med Cell Longev.

## 1. Introduction

Approximately 5% of breast cancers are metastatic at diagnosis, and 20-30% of localized breast cancers become metastatic [1]. The median survival of metastatic breast cancer ranges from two to three years with five-year survival rates of 25% [2]. Physical activity may be beneficial to breast cancer survivors and has been inversely associated with breast cancer recurrence and mortality [3, 4]. However, little is known regarding the effect of physical activity in patients with metastatic breast cancer.

Several biological pathways may explain the beneficial effect of physical activity on breast cancer progression or recurrence, including an effect on levels of sex hormones, mediators of inflammation, insulin resistance, and antioxidant pathways. Although acute physical exercise is known to increase oxidative stress temporarily, regular training reduces basal levels of oxidative stress, particularly by increasing enzymatic antioxidant defenses [5]. In this context, the improvement of the antioxidant enzyme efficiency by PA may be protective in breast cancer and, more specifically, in metastatic breast cancer. Antioxidant enzymes could neutralize the overproduction of ROS resulting from metastases as increased plasma DNA repair and antioxidant capacities during chemotherapy significantly improved the survival rates of metastatic breast cancer patients [6, 7]. Several randomized trials have demonstrated the beneficial effects of physical activity on oxidative stress status in several diseases including breast cancer [8]. To our knowledge, no previous PA intervention study has been conducted that examined the change in oxidative stress markers in patients with metastatic breast cancer.

Damages to DNA, lipids, and proteins by reactive oxygen species (ROS) (DNA oxidation and lipid and protein peroxidation, respectively) are commonly used measures of oxidative stress. The oxidation of DNA is known to play a significant role in carcinogenesis [9], tumor promotion [10], and breast cancer recurrence [11]. In addition, chemotherapy likely induces oxidative damage [12]. 8-Hydroxy-2′-deoxyguanosine (8-OHdG), the most frequently studied DNA oxidation marker, has been shown to predict breast cancer risk [13], and higher 8-OHdG levels have been observed in the plasma of breast cancer patients compared to controls [14]. Metastatic progression of human breast cancers has been associated with hydroxyl radical-induced DNA damage [15]. Moreover, markers of lipid peroxidation increase breast cancer risk [16] and decrease prognosis [17]. Similarly to 8-OhdG, plasma lipid and protein oxidation markers (malondialdehyde [MDA] and advanced oxidation protein products [AOPP], respectively) were statistically significantly higher in patients with breast cancer compared to controls [18]. Interestingly, plasma lipid oxidation is also higher in metastatic than in localized breast cancer [19]. In contrast, antioxidants may protect from breast cancer by neutralizing the overgenerated ROS [20]; however, the antioxidant defense mechanisms are weakened in breast cancer patients [20]. Specifically, superoxide dismutase (SOD) catalyzes the dismutation of superoxide anion into hydrogen peroxide that is subsequently detoxified by catalase or glutathione peroxidase (GPX) [21]. Case-control studies have observed an association between impaired oxidant to antioxidant balance and breast cancer [22, 23], including breast cancer prognosis [24, 25]. Although the role of oxidative stress in carcinogenesis and metastatic expansion has already been shown *in vitro* or in animal models, its role as a biomarker of the disease progression is still unknown.

The article "Impact of Physical Activity on Oxidative Stress Markers in Patients with Metastatic Breast Cancer" was published in 2021. Journal: Oxid Med Cell Longev.

The present study was performed as a secondary objective of the ABLE Single-Arm Feasibility Trial [26]. The purpose of this analysis was to generate preliminary data on the association between physical activity, oxidative stress, and clinical disease outcomes in a group of metastatic breast cancer participants of the ABLE Trial. The specific objectives were to evaluate in this six-month physical activity intervention: (1) the change in oxidative stress biomarker levels after the intervention, (2) the associations between oxidative stress biomarkers and physical activity levels, and (3) the associations between oxidative stress biomarkers at baseline and clinical outcomes (including metastatic progression) during the intervention.

## 2. Methods

### 2.1. Study Design

The ABLE Trial was a single-arm intervention trial based on a six-month, home-based, unsupervised, and personalized physical activity program in women newly diagnosed with metastatic breast cancer, conducted in the Léon Bérard Comprehensive Cancer Center (Lyon, France). Methodology and results of ABLE Trial have been described in details elsewhere [26, 27]. The study protocol was approved by the local research ethics committee (*Comité de Protection des Personnes Sud-Est IV*), and the study database was reported to the National Commission for Data Protection and Liberties (CNIL; reference number: 1994192). The ABLE Trial was registered on http://www.clinicaltrials.gov (NCT number: NCT03148886).

The article "Impact of Physical Activity on Oxidative Stress Markers in Patients with Metastatic Breast Cancer" was published in 2021. Journal: Oxid Med Cell Longev.

### 2.2. Study Participants, Inclusion, and Follow-Up

Patients recruited were female, 18 to 78 years old, newly diagnosed with a primary or secondary metastatic breast cancer histologically confirmed within the last three months, and treated in the cancer center by chemotherapy, radiotherapy, hormonal therapy, and/or targeted therapy. They had an Eastern Cooperative Oncology Group (ECOG) performance status < 2, were French speaking, and were able to complete questionnaires and follow instructions in French and had a valid health insurance plan. Certification from their treating oncologist of no contraindications to physical activity was required for patients volunteering to participate in the study. Exclusion criteria were having untreated brain metastases, pregnancy, or contraindications to physical activity (e.g., uncontrolled hypertension, cardiac disease). All patients gave a written informed consent prior to their entry into the study.

Assessments were conducted at baseline, at the end of the intervention at six-month, and again at 13-month (i.e., seven-month postintervention) follow-up to assess tumor progression and mortality outcomes of all participants.

### 2.3. Physical Activity Intervention

The intervention was a six-month, home-based, unsupervised, and personalized physical activity program based on a daily step recommendation as previously described [27, 28]. Patients were asked to wear a physical activity tracker (Nokia Go wristband, Nokia, France) starting at entry into the study and throughout the six-month duration of the intervention. The physical activity prescription was individualized to each participant and provided to them by the study exercise trainer. It was based on their physical fitness and the average number of steps that were recorded during the week prior to the intervention. The prescription was a goal of steps per day that was updated biweekly during the intervention based on their activity. The step target was increased by a maximum of 1000 steps per week up to a maximum of 10,000 steps at which point the participants were asked to maintain this level of physical activity. When participants experienced any difficulty reaching their target number of steps per day because of issues related to their treatment, illness, or other factors, the target could be lowered after discussion between the exercise trainer and the participant.

### 2.4. Data Collection

#### 2.4.1. Clinical and Anthropometrical Characteristics

Clinical data were recorded throughout the study and extracted from the participants' electronic medical records. They included personal history of breast cancer, sites and number of metastases, current treatment, presence of comorbidities (cardiac, respiratory, metabolic, and neurologic), and blood count. The Response Evaluation Criteria in Solid Tumors (RECIST) was used to assess tumor progression between diagnosis and the end of the physical activity program. Anthropometrics were assessed at baseline and at six-month and included measured standing height (cm) and body weight (kg) and calculated body mass index (BMI; kg/m^2^).

The article "Impact of Physical Activity on Oxidative Stress Markers in Patients with Metastatic Breast Cancer" was published in 2021. Journal: Oxid Med Cell Longev.

#### 2.4.2. Physical Fitness Tests

Distance of the six-minute walk test was measured as the maximum walking distance on a 30-meter-long flat corridor during six minutes. Isometric maximal strength of the dominant leg extensors was measured with a dynamometer (DFS II Series Digital Force Gauges, Chatillon, Florida, United States). The number of steps per day was measured with an activity tracker (Nokia Go® wristband, Nokia France, Issy-les-Moulineaux, France) and regularly downloaded through the activity tracker smartphone application (Nokia Health Mate®).

#### 2.4.3. Physical Activity Level

Physical activity level was evaluated by the French version of the long form of International Physical Activity Questionnaire (IPAQ) and measured in metabolic equivalent of task (MET)-minutes/week [29]. Sedentary activities were assessed using sitting time—in minutes/week—measured by the IPAQ questionnaire.

#### 2.4.4. Blood Biological Data

A fasting 7 mL blood sample was collected at baseline and at the end of the six-month intervention. Blood samples were drawn into ethylenediaminetetraacetic acid (EDTA) blood collection tubes, centrifuged at 800*g* for 10 minutes. Plasma and buffy coat were aliquoted into cryotubes that were immediately frozen to -80°C until analysis that occurred between 1 and 19 months after sampling. Each participant's samples were analyzed in the same run/experiment to avoid interassay variability. From the buffy coat, leukocytes were isolated from other blood cells by washing them three times in sterile PBS by centrifugation at 3400*g* at 4°C for 10 min. Protein concentration of leucocyte samples was assayed with a BCA kit (Novagen #71285.3, Darmstadt, Germany), and all data from leucocytes were normalized by milligrams of total protein. All spectrophotometry and fluorometry measurements were performed with a TECAN Infinite 2000 plate reader (Männedorf, Switzerland) as previously published [30] and briefly described below.

#### 2.4.5. Plasma Antioxidant Enzyme Activities: Catalase, Glutathione Peroxidase (GPX), and Superoxide Dismutase (SOD)

Plasma catalase activity was determined by measuring the kinetics of formaldehyde appearance formed by the reaction between methanol and hydrogen peroxide (H_2_O_2_) and revealed by Purpald solution. Formaldehyde concentration was measured spectrophotometry at 540 nm.

The article "Impact of Physical Activity on Oxidative Stress Markers in Patients with Metastatic Breast Cancer" was published in 2021. Journal: Oxid Med Cell Longev.

Plasma GPX activity was determined by measuring the kinetics of nicotinamide adenine dinucleotide phosphate hydrogen (NADPH) consumption at 340 min in the presence of H_2_O_2_, glutathione reductase, and reduced glutathione.

Plasma SOD activity was determined by the degree of inhibition of the reaction between superoxide radicals, produced by a hypoxanthine-xanthine oxidase system, and nitroblue tetrazolium (NTB) producing formazan blue. The kinetics of formazan blue appearance was measured at 560 nm.

#### 2.4.6. Prooxidant Enzyme Activities: NADPH Oxidase (NOX) and Myeloperoxidase (MPO)

Leucocyte NOX activity was determined by measuring at 560 nm the kinetics of formazan blue appearance in the presence of NTB and NADPH. For this assay, 1 mM of NaCN was added into all the plasma samples to inhibit SODCu-Zn.

MPO activity was measured in plasma as well as in leucocytes by the determination of the kinetic absorbance at 653 nm after addition of H_2_O_2_ and 3,3′,5,5′-tetramethylbenzidine (TMB).

#### 2.4.7. Oxidative Stress Damage Markers: Advanced Oxidation Protein Products, Malondialdehyde, and DNA Oxidation (8-Hydroxy-2′-Deoxyguanosine: 8-OHdG)

Plasma AOPP concentration was measured at 340 nm by the addition of acetic acid using chloramine-T in the presence of potassium iodide as standard.

Plasma MDA concentration was determined after addition of 2-thiobarbituric acid (TBA) and HCl. The complex formed by MDA with TBA at 100°C was measured by spectrophotometry at 532 nm using 1,1,3,3-tetraethoxypropane as standard.

Plasma 8-OHdG concentration was measured using an ELISA kit assay (AS15 2887, Agrisera, Vännäs, Sweden).

### 2.5. Statistical Analysis

Participants' characteristics were described using means and standard deviations (SDs) for quantitative data and frequencies and percentages for qualitative data. Correlations between biomarkers, physical fitness, and physical activity were estimated using the Spearman correlation coefficient.

The change in oxidative stress biomarkers level after the six-month physical activity intervention was assessed using the Wilcoxon signed-rank test. The associations between oxidative stress biomarkers at baseline and clinical outcomes including death and metastatic progression were analyzed by Kruskal-Wallis test. Data were analyzed using the SAS software (version 9.4., SAS Institute Inc., Cary, NC, USA).

## 3. Results

Baseline characteristics of the study population have been previously described [28]. Briefly, there were 49 participants in the ABLE Trial recruited between October 2016 and July 2017 and followed up until January 2018. The participants had a mean age (±SD) of 55 (±10) years and a mean BMI of 26.08 ± 5.78 kg/m^2^, and 53% were considered overweight or obese at inclusion (Table 1). Most of the participants experienced a metastatic breast cancer recurrence (71.4%) and received first-line hormone therapy for their metastatic breast cancer (55.1%).

The article "Impact of Physical Activity on Oxidative Stress Markers in Patients with Metastatic Breast Cancer" was published in 2021. Journal: Oxid Med Cell Longev.

Detailed results regarding the clinical outcomes (deaths, RECIST metastatic progression), physical fitness, and physical activity level have been previously reported [28]. In brief, among the 49 patients, seven had metastatic progression during the study according to RECIST criteria, four died before the end of the intervention, and five died during the subsequent follow-up (Table 2). 96% of the patients adhered to the physical activity prescription (attrition rate 2%). Both the six-minute walking distance (+7%, *p* < 0.001) and isometric maximal strength of quadriceps (+22%, *p* < 0.001) tests increased significantly between baseline and the end of the six-month intervention. Their physical activity levels remained stable between baseline and the end of the intervention (*p* = 0.66); however, sitting time decreased significantly (*p* < 0.01) during the same period and BMI levels decreased (-2.7%, *p* < 0.05).

### 3.1. Oxidative Stress, Prooxidant Markers, and Antioxidant Markers at Baseline and at the End of the Six-Month Intervention

Overall, plasma GPX activity (+17%, *p* = 0.04) and plasma MDA concentration (+9%, *p* = 0.03) significantly increased between baseline and the end of the intervention (Figure 1). All other plasma and leucocyte markers (SOD, NOX, MPO, AOPP, CAT, and 8OHdG) did not change statistically significantly during the intervention (Table 3).

### 3.2. Associations between Oxidative Stress, Prooxidant Markers, and Antioxidant Markers, and Physical Fitness Tests, Physical Activity, and BMI at Baseline

At baseline, physical activity level (IPAQ score) was positively correlated with plasma GPX (*r* = 0.39; *p* = 0.01) and negatively correlated with NOX activity in the leucocytes (*r* = −0.39; *p* = 0.01). The number of daily steps was positively correlated with plasma GPX activity (*r* = 0.49; *p* = 0.01). Isometric maximal strength of quadriceps was negatively inversely correlated with plasma MDA (*r* = −0.31; *p* = 0.04). At baseline, patients below the 630 MET-min/week recommended level of physical activity had lower plasma GPX activity (-30%, *p* = 0.02) and higher NOX activity in the leucocytes (+10%, *p* = 0.04). At baseline, BMI was not significantly correlated with any of the plasma and leucocyte oxidative stress, prooxidant markers, and antioxidant markers except with plasma SOD (*r* = 0.33; *p* = 0.018). BMI at baseline was positively correlated with increase (end of intervention minus baselines) in OHdG concentration during the six-month intervention (*r* = 0.32; *p* = 0.03). The correlations between changes (end of intervention minus baseline) of oxidative stress, prooxidant markers and antioxidant markers, and physical fitness tests and physical activity are presented in Figure 2.

The article "Impact of Physical Activity on Oxidative Stress Markers in Patients with Metastatic Breast Cancer" was published in 2021. Journal: Oxid Med Cell Longev.

Overall, two important results are noteworthy. First, the change of GPX activity was strongly and positively correlated (indicated by the magnitude of blue circles) with changes in physical fitness and activity levels (i.e., IPAQ, daily step number, and six-minute walking distance). Second, changes of NOX leucocyte activity were strongly and negatively correlated (indicated by the magnitude of red circles) with changes in physical activity and fitness level.

More specifically, the changes of plasma GPX activity were positively correlated with changes of daily step number (*r* = 0.49; *p* = 0.01) and physical activity level (IPAQ score) (*r* = 0.39; *p* < 0.01). The changes of NOX activity in leucocytes and physical activity level (IPAQ score) were negatively correlated (*r* = −0.39; *p* < 0.01). The changes in AOPP concentration and sedentary time during the six-month intervention were negatively correlated (*r* = 0.33; *p* = 0.03). Changes of isometric maximal strength of quadriceps and plasma MDA concentration were negatively correlated (*r* = −0.31; *p* = 0.04). The changes of the six-minute walking distance were negatively correlated with changes of plasma SOD (*r* = −0.32; *p* = 0.03) and catalase activities (*r* = −0.40; *p* < 0.01).

### 3.3. Biomarkers of Oxidative Stress at Baseline Are Associated with Clinical Outcomes during the Six-Month Intervention

Participants who had RECIST metastatic progression or who died during the intervention period had statistically significantly higher plasma MDA concentrations (+20%, *p* = 0.04) and lower plasma AOPP concentrations (-46%, *p* = 0.01) at baseline compared to patients without metastatic progression (Table 4). There were no other differences at baseline for the other biomarkers for participants with RECIST metastatic progression or who died during the intervention period and those that did not.

## 4. Discussion

To our knowledge, this ancillary study of the ABLE Trial is the first to examine the change in blood oxidative stress status during a six-month physical activity intervention in women with metastatic breast cancer. The three main findings from this analysis were (1) plasma GPX activity and plasma MDA increased statistically significantly after the six-month physical activity program, (2) AOPP was identified as a favorable and MDA as unfavorable biomarkers because they are associated with metastatic breast cancer progression according to death and RECIST criteria, and (3) plasma GPX activity was positively correlated with physical activity and fitness levels and negatively correlated with changes of plasma NOX activity and physical activity and fitness levels.

The article "Impact of Physical Activity on Oxidative Stress Markers in Patients with Metastatic Breast Cancer" was published in 2021. Journal: Oxid Med Cell Longev.

As previously reported in studies with other chronic diseases [31, 32] and in breast cancer participants [7], the increase in plasma GPX activity observed between baseline and the end of the intervention could be attributed to the physical activity intervention. This hypothesis is supported by several observations in our study. These include the positive associations between plasma GPX activity and physical activity level and daily number of steps at baseline, the higher GPX activity for participants who reached the recommendations of physical activity over 630 MET-min/weeks, and more importantly, the positive associations between changes GPX activity and physical activity and fitness. It could be hypothesized that the increase in GPX activity during physical activity could favor a reduction in cellular and circulating ROS content. Indeed, ROS are known to play a role in breast cancer recurrence and metastasis; in particular, the radical hydroxyl suggested to be involved in the metastatic progression of human breast cancer [15].

In contrast to GPX activity, the prooxidant enzyme NOX activity in the leucocytes was negatively associated with the physical activity level (IPAQ score) at baseline, and more importantly, leucocyte NOX activity changes are negatively associated with changes in physical activity and fitness (Figure 2). NOX being involved in the superoxide production, physical activity level may protect from ROS production via the NOX pathway as it has been shown recently in healthy subjects [33]. Many mechanisms have been described to explain the downregulation of NOX activity by regular physical activity [34]; however, the reduction of fat tissue during physical activity intervention might be the most plausible since obesity upregulates the systemic expression of NOX [35]. The decrease in BMI that we observed in our population during the six-month physical activity intervention may support this latter hypothesis. Indeed, decrease in obesity by low-intensity physical intervention reduced systemic oxidative stress, particularly [36].

Overall, these correlations between changes in GPX activity, NOX activity, and physical activity and fitness suggest that plasma GPX and leucocyte NOX activities could be relevant biomarkers of physical activity and fitness changes in the context on metastatic breast cancer.

The article "Impact of Physical Activity on Oxidative Stress Markers in Patients with Metastatic Breast Cancer" was published in 2021. Journal: Oxid Med Cell Longev.

MDA concentration was negatively associated with the isometric maximal strength of quadriceps at baseline. These results should be considered in relation to the significant improvement of isometric maximal strength of quadriceps observed during the six-month intervention, the maintenance of the physical activity level (IPAQ score), and the decrease in the sedentary time after the intervention [28]. The increase in MDA concentration observed between baseline and the end of the six-month intervention may be attributable to the disease progression [11] and anticancer treatment [12] specific to our population that may mask the effect of the physical activity intervention. Higher plasma MDA concentration at baseline in participants with tumor progression or who died during the six-month intervention suggests that plasma MDA could be an unfavorable biomarker for metastatic breast cancer participants undergoing a physical activity intervention. In contrast, concentration of plasma AOPP, an advanced oxidation protein product, was significantly lower for participants with tumor progression or who died during the six-month intervention and might be considered as favorable biomarker in this population. Although AOPP and MDA are two markers of oxidative stress, they are not produced from the same pathway and thus may explain why the effect was opposite regarding their associations with death and tumor progression. MDA is an end-product of polyunsaturated fatty acid oxidation [37], and AOPP results from the activation of the MPO pathway in the circulating immune cells [38]. Hence, plasma MDA may result from the oxidation of cell membranes by ROS. On the contrary, AOPP may induce the activation of antioxidant enzyme molecular pathways since oxidized proteins have been suggested to play a significant role in the antioxidant cell signaling. In our context, higher AOPP concentration in those who did not progress and died could favor biological processes limiting the cellular tumor development.

The changes in 8OHdG concentration and sedentary time during the six-month intervention were positively correlated. This result shows that, in breast cancer participants undergoing a physical activity program, a reduction of sedentary behavior may lead to attenuation of the oxidative-inflammatory loop leading to various chronic diseases [39].

Interestingly, it was shown that BRCA1 may be required for DNA repair so important in breast cancer development [40]. More specifically, an in vitro study reported that BRCA1 was associated to unpaired antioxidant capacity [41]. In this context, it was shown that breast cancer participants with the BRCA1 mutation presented a higher degree of oxidative damage to lipids (8-isoprostane and MDA) but not AOPP in the saliva [42]. In our study, only two patients presented BRCA1 mutation; it is thus unlikely that this mutation was involved in the oxidative stress response of our patients.

The article "Impact of Physical Activity on Oxidative Stress Markers in Patients with Metastatic Breast Cancer" was published in 2021. Journal: Oxid Med Cell Longev.

Several study limitations should be considered. First, the ABLE Trial was not powered to detect changes for oxidative stress outcomes and the sample size was too small to detect statistically significant changes in plasma 8OHdG concentration. Contrary to what was expected, plasma 8OHdG was not statistically significantly associated with physical activity and physical fitness or with disease progression outcomes (metastasis progression and deaths). Second, the study design used for ABLE Trial was intentionally a single-arm intervention. The *per se* effects of disease progression and pharmacological treatments versus the physical activity intervention on the oxidative stress status cannot be differentiated. Nevertheless, it is likely that lipid peroxidation and DNA oxidation markers would increase with time and antioxidant enzyme would decrease in metastatic breast cancer patients [6, 19]. Hence, these results will have to be confirmed in larger randomized controlled trial. Third, the physical activity intervention was home-based, unsupervised, and personalized. This kind of intervention could have influenced the magnitude of blood oxidative stress response [43] since it induced heterogeneous physical activity among the participants with respect to time and intensity of the activity done.

## 5. Conclusion

These results provide some preliminary evidence for a role of oxidative stress and antioxidant enzymes in the association of physical activity with outcomes for metastatic breast cancer. They also suggest that plasma AOPP could be a favorable biomarker and MDA an unfavorable one for metastatic breast cancer patients. The clinical relevance of these biomarkers as prognostic factors in metastatic breast cancer patients requires confirmation in a larger cohort follow-up. Our ongoing national, multicenter, randomized controlled ABLE02 Trial has been designed to address some of the limitations of this trial and will assess the efficacy of a physical activity program in women with metastatic breast cancer [44].

## Figures and Tables

**Figure 1:** Change of MDA (a) and GPX (b) between baseline and the end of the six-month physical activity intervention, ABLE study, 2016-2018. MDA: malondialdehyde; GPX: glutathione peroxidase. ^∗^*p* < 0.05 vs. baseline.

The article "Impact of Physical Activity on Oxidative Stress Markers in Patients with Metastatic Breast Cancer" was published in 2021. Journal: Oxid Med Cell Longev.

**Figure 2:** Correlation plot of changes in oxidative stress markers, physical activity level, and physical fitness between baseline and the end of the six-month physical activity intervention, ABLE study, 2016-2018. CAT: catalase; SOD: superoxide dismutase; NOX: nicotinamide adenine dinucleotide phosphate oxidase; MPO: myeloperoxidase; 8-OhdG: 8-hydroxydeoxyguanosine; AOPP: advanced oxidation protein products; MDA: malondialdehyde; GPX: glutathione peroxidase; 6WD: 6-minute walking distance; Quadriceps: isometric quadriceps strength; PA: total physical activity; Daily steps: mean steps per day over a month. Blue and red circles represent positive and negative correlations, respectively; size and color intensity of the circle represent the strength of the correlation.

**Table 1:** Demographic baseline clinical characteristics of women with metastatic breast cancer, ABLE Trial, Lyon, France, 2016-2018.

Baseline characteristics	All participants (*n* = 49)
Age (year), mean (SD)	54.91 (10.41)
Anthropometrics	
Height (m), mean (SD)	1.62 (0.06)
Weight (kg), mean (SD)	69.12 (15.71)
BMI (kg/m^2^), mean (SD)	26.08 (5.78)
Underweight (<18.5 kg/m^2^), *n* (%)	3 (6.1%)
Normal weight (<25 kg/m^2^), *n* (%)	20 (40.8%)
Overweight (25–30 kg/m^2^), *n* (%)	16 (32.7%)
Obese (>30 kg/m^2^), *n* (%)	10 (20.4%)
Clinical	
Number of metastatic localizations, *n* (%)	4.65 (3.05)
De novo metastatic breast cancer, *n* (%)	14 (28.6%)
Hormone therapy, n (%)	27 (55.1%)
Chemotherapy, *n* (%)	22 (44.9%)
Histological subtype	
HER2+	1 (2.0%)
Luminal A	29 (59.2%)
Luminal B	6 (12.2%)
Triple negative	13 (26.5%)
Number of metastatic locations	4.65 (3.05)
Metastatic locations	
Cerebral	6 (12.2%)
Bone	33 (67.3%)
Lung	15 (30.6%)
Nodes	24 (49.0%)
Skin	1 (2.0%)
Liver	12 (24.5%)
Other	20 (40.8%)
Blood count	
Hemoglobin (g/dL)	12.88 (1.48)
Creatinine (*μ*mol/L)	60.67 (11.79)
Alanine aminotransferase (UI/L)	25.39 (15.98)
Aspartate aminotransferase (UI/L)	28.51 (16.63)
Alkaline phosphatase (UI/L)	109.25 (82.40)
Gamma-glutamyl transpeptidase (UI/L)	71.58 (94.06)
Comorbid conditions	
Cardiac disease	17 (34.7%)
Metabolic	12 (24.5%)
Respiratory	4 (8.2%)
Neurologic	1 (2.0%)

BMI: body mass index.

**Table 2:** Change in physical activity level, physical fitness, ABLE Trial, 2016-2018.

	Baseline (*n* = 49)	After 6 months (*n* = 45)	*p* ^a^
Physical activity level			
Total physical activity (MET-minutes/week) (mean, SD)	2031.3 (2213.1)	1940.8 (1762.4)	0.66
Achieving physical activity recommendations, *n* (%)	34 (69.4%)	34 (77.3%)	0.26
Mean steps per day over a month (mean, SD)	5592.9 (4064.2)	5398.7 (3888.2)	0.28
Sitting time (MET-min/week)	538.5 (221.3)	483.0 (227.1)	**<0.01**
Physical fitness			
6-minute walking distance (m), mean (SD)	451.6 (99.7)	482.6 (106.2)	0.85
Handgrip strength, right side (kg), mean (SD)	26.2 (6.1)	26.2 (4.3)	0.17
Handgrip strength, left side (kg), mean (SD)	30.11 (35.33)	24.06 (4.39)	0.25
Isometric quadriceps strength (*N*), mean (SD)	194.2 (69.1)	236.4 (78.6)	**<0.01**
Body mass index (kg/m^2^)	26.1 (5.8)	25.4 (5.8)	**0.03**

^a^Wilcoxon signed-rank test.

The article "Impact of Physical Activity on Oxidative Stress Markers in Patients with Metastatic Breast Cancer" was published in 2021. Journal: Oxid Med Cell Longev.

**Table 3:** Change in antioxidant, prooxidant enzymes, and oxidative stress markers, ABLE Trial, 2016-2018.

Biomarkers	Baseline (*n* = 49)	After 6 months (*n* = 45)	*p* ^a^
Antioxidant enzymes			
CAT (*μ*mol.min^−1^.L^−1^), mean (SD)	34.14 (18.66)	37.85 (18.70)	0.40
SOD (*μ*mol.min^−1^.L^−1^), mean (SD)	9.17 (4.31)	9.00 (4.59)	0.54
Prooxidant enzymes			
NADPH oxidase leucocytes (*μ*mol.min^−1^.mg^−1^ of protein), mean (SD)	0.22 (0.06)	0.22 (0.06)	0.89
MPO plasma (*μ*mol.min^−1^.L^−1^), mean (SD)	114.07 (58.03)	121.75 (51.49)	0.29
MPO leucocytes (*μ*mol.min^−1^.mg^−1^ of prot), mean (SD)	15.90 (4.38)	15.76 (7.86)	0.74
Oxidative stress markers			
8-OHdG (*μ*g.L^−1^), mean (SD)	17.13 (18.16)	17.72 (15.42)	0.46
AOPP (*μ*mol.L^−1^), mean (SD)	78.96 (55.20)	87.37 (55.88)	0.44

^a^Wilcoxon signed-rank test. CAT: catalase; SOD: superoxide dismutase; NADPH: nicotinamide adenine dinucleotide phosphate; MPO: myeloperoxidase; 8-OhdG: 8-hydroxydeoxyguanosine; AOPP: advanced oxidation protein products.

**Table 4:** Antioxidant, prooxidant enzymes, and oxidative stress markers at baseline between patients with unfavorable and favorable clinical outcomes, ABLE Trial, 2016-2018.

Biomarkers	Favorable outcomes (*n* = 38)	Unfavorable outcomes (*n* = 11)	*p* ^a^
Antioxidant enzymes			
CAT (*μ*mol.min^−1^.L^−1^), mean (SD)	34.32 (18.94)	33.55 (18.54)	0.87
GPX (*μ*mol.min^−1^.L^−1^), mean (SD)	70.55 (25.48)	63.17 (20.19)	0.22
SOD (*μ*mol.min^−1^.L^−1^), mean (SD)	9.62 (4.20)	7.69 (4.56)	0.28
Prooxidant enzymes			
NADPH oxidase leucocytes (*μ*mol.min^−1^.mg (prot)^−1^), mean (SD)	0.22 (0.05)	0.24 (0.07)	0.40
MPO plasma (*μ*mol.min^−1^.L^−1^), mean (SD)	111.59 (57.83)	122.41 (60.72)	0.37
MPO leucocytes (*μ*mol.min^−1^.mg(prot)^−1^), mean (SD)	15.78 (4.22)	16.31 (5.09)	0.58
Oxidative stress markers			
MDA (*μ*mol.L^−1^), mean (SD)	11.04 (2.96)	13.33 (3.66)	**0.04**
8-OHdG (*μ*g.L^−1^), mean (SD)	17.67 (18.99)	15.33 (15.71)	0.55
AOPP (*μ*mol.L^−1^), mean (SD)	88.07 (59.63)	48.31 (13.34)	**0.008**

^a^Kruskal-Wallis test. CAT: catalase; SOD: superoxide dismutase; NADPH: nicotinamide adenine dinucleotide phosphate; MPO: myeloperoxidase; 8-OhdG: 8-hydroxydeoxyguanosine; AOPP: advanced oxidation protein products; MDA: malondialdehyde; GPX: glutathione peroxidase. Unfavorable clinical outcomes: RECIST metastatic progression or death during the intervention period. Favorable clinical outcomes: no RECIST metastatic progression and no death during the intervention period.

The article "Impact of Physical Activity on Oxidative Stress Markers in Patients with Metastatic Breast Cancer" was published in 2021. Journal: Oxid Med Cell Longev.

## Data Availability

The data used to support the findings of this study are available from the corresponding author upon request.
